This article has been retracted.

# Investigation on Risk Stratification and the Prognostic Value of hs-TnT Combined with MMP-2 in Patients with Acute Coronary Syndrome

**DOI:** 10.1155/2021/1040171

**Published:** 2021-11-23

**Authors:** Ying Li, Li Li, Kun Wang, Pengtao Wu, Yijie Cui

**Affiliations:** ^1^The No.2 Hospital of Baoding Physical Medicine and Rehabilitation Department, Baoding, 071000 Hebei, China; ^2^The No.2 Hospital of Baoding Internal Medicine and Cardiovascular Department, Baoding, 071000 Hebei, China; ^3^The No.2 Hospital of Baoding Computerized Tomography Scan Room, Baoding, 071000 Hebei, China

## Abstract

**Objective:**

The aim of this study was at investigating the risk stratification and prognostic value of hypersensitive troponin T (hs-TnT) combined with matrix metalloproteinase 2 (MMP-2) in patients with acute coronary syndrome (ACS).

**Methods:**

80 patients with coronary syndrome admitted to our hospital from January 2019 to January 2020 and 40 healthy people (control group) in the same period were selected. According to different types of diseases, the patients were divided into an acute group (*n* = 40) and stable group (*n* = 40). Besides, they all were monitored by the hs-TnT value, serum MMP-2, and coronary angiography at admission and the comparative analysis was carried out. The patients in both groups were followed up for 30 days, and the incidence of adverse cardiovascular events in the patients during this period was recorded.

**Results:**

Compared with those in the control group, the MMP-2 and hs-TnT levels in the acute group and the stable group were significantly higher and the MMP-2 and hs-TnT levels in the acute group were significantly higher than those in the stable group, with statistically significant differences (*P* < 0.05). The 30-day follow-up results showed that the incidence of adverse cardiovascular events in the acute group was significantly higher than that in the stable group, with statistically significant differences (*P* < 0.05). The hs-TnT and MMP-2 levels in the acute myocardial infarction (AMI) group were significantly higher than those in the unstable angina pectoris (UAP) group, with statistically significant differences (*P* < 0.01). The hs-TnT and MMP-2 levels in the non-single-vessel group were significantly higher than those in the single-vessel group, with statistically significant differences (*P* < 0.01).

**Conclusion:**

The hs-TnT and MMP-2 high expression levels are closely associated with myocardial injury, and they can effectively predict the severity of patients' disease. In addition, the hs-TnT and MMP-2 elevated levels can be considered as an important index to judge the short-term treatment efficacy and the risk stratification of early ACS, playing an important role in clinical treatment and rehabilitation in the later stage.

## 1. Introduction

Acute coronary syndromes (ACS) represent a major cause of mortality in our country. Currently, there is a very wide spectrum of clinical presentation since the actual classification of ACS is based on electrocardiographic presentation, that is, to say based on the absence or presence of ST segment elevation. Most patients with acute coronary syndrome (ACS) present with chest pain and a few with upper abdominal pain [1]. Medically, ACS is divided into non-ST-segment elevation ACS and ST-segment elevation ACS [2–4]. This disease is caused by increased blood viscosity and myocardial oxygen consumption, as well as sympathetic excitation, thus resulting in the rupture or erosion of unstable atherosclerotic plaque, massive platelet aggregation, and even thrombosis. Non-ST-segment elevation ACS mostly occurs at night or at rest and lasts for more than 20 minutes. A diagnosis of ACS should be considered in all patients presenting with ischemic symptoms. Clinical signs and symptoms of ischemia include various combinations of chest pain; upper extremity, mandibular, or epigastric discomfort; dyspnea; diaphoresis; nausea; fatigue; or syncope. The pain and discomfort associated with an ACS event may occur with exertion or at rest and are often diffuse rather than localized [5].

Besides, the manifestation of this disease is radiation chest pain, accompanied by burning and a sense of pressure, and some patients also present with chest distress and sense of being close to death [6]. Generally speaking, ACS has the characteristics of acute onset and rapid progress, which seriously endangers patients' health and life. Therefore, when the patients have the above suspected symptoms, they should see a doctor immediately to avoid delaying treatment. With the advancement of the medical level, it has been found that hypersensitive troponin has a significant clinical value for the diagnosis of ACS [7]. At present, the main diagnostic criteria for this disease are the global definition of myocardial infarction whose core is the elevation of myocardial markers, namely, the elevation of troponin.

As one of the matrix metalloproteinase genes, MMP-2 is widely distributed in the human body and most of the cells including endothelial cells, epithelial cells, and stromal cells are expressed. MMP-2 causes the rupture of plaque cells to a certain extent mainly by degrading the extracellular matrix of plaque, as well as digesting and destroying the fibrous structure, and finally leads to ACS [8]. Therefore, in order to further investigate the risk stratification and prognostic values of hypersensitive troponin T (hs-TnT) combined with MMP-2 in patients with ACS, 80 patients with coronary syndromes admitted to our hospital from January 2019 to January 2020 and 40 healthy people in the same period were selected as study objects and the summary report is as follows.

## 2. Materials and Methods

### 2.1. General Information

In this study, 80 patients with coronary syndromes admitted to our hospital from January 2019 to January 2020 and 40 healthy people in the same period were selected as study objects. According to different types of diseases, patients were divided into the acute group and stable group. Among them, there were 19 males and 21 females both aging from 37 to 73 years in the acute group, with an average age of 53.27 ± 1.45 years, and their course of disease ranged from 1 to 6 years, with an average course of disease of 3.05 ± 0.56 years. The coronary angiography showed that 18 patients had single-vessel disease and 22 patients had non-single-vessel (two or more) disease. Among them, 26 patients had acute myocardial infarction (AMI) and 14 patients had unstable angina pectoris (UAP). There were 18 males and 22 females aging from 39 to 71 years in the stable group, with an average age of 53.04 ± 1.38 years, and their course of disease ranged from 2 to 8 years, with an average course of disease of 3.21 ± 0.63 years. The coronary angiography also revealed that 23 patients had single-vessel disease and 17 patients had non-single-vessel disease. Among them, 25 patients had AMI and 15 patients had UAP. There were 20 males and 20 females aging from 37 to 68 years in the control group, with the average age of 52.85 ± 1.46 years. There were no significant differences in age, sex ratio, and other general data among the three groups (*P* > 0.05), with research significance. This study was approved by the Hospital Ethics Committee, and the patients and their families were informed of the purpose and process of this study and signed the informed consent.

### 2.2. Inclusion Criteria

According to the classification criteria of International Society of Federation of Cardiology and World Health Organization on acute myocardial infarction and stable angina pectoris, the patients were divided into the acute group, stable group, and control group. Among them, the control group with healthy people undergoing physical examination in the same period had normal results of electrocardiogram (ECG) and coronary angiography without coronary heart disease.

### 2.3. Exclusion Criteria

Patients had renal and hepatic dysfunction, were allergic to iodine, had myocardial infarction and trauma or underwent surgery recently, had malignant tumors, and had arrhythmia and atrial fibrillation.

### 2.4. Methods

#### 2.4.1. Clinical Data Collection

The age, gender, drinking and smoking history, triglyceride, hyperlipidemia, and hypertension of patients were included.

#### 2.4.2. Sample Collection, Processing, and Preservation

Serum samples were collected from all the patients. 10 ml of fasting venous blood was collected from the three groups and placed in anticoagulant tubes. Blood centrifuge (manufacturer: Guangzhou Jidi Instrument Co. Ltd.; model type: JIDI-4D-WS) was adopted to centrifuge at 3000 r/min for 10–15 min. Then, the supernatants were taken and stored at −75°C for use. Enzyme-linked immunosorbent assay was adopted by an experienced technician to detect the MMP-2 expression levels in serum, and chemiluminescence immunoassay was also carried out to determine the hs-TnT expression levels of patients. The serum MMP-2 kit was provided by Shanghai Bairui Biological Technology Co. Ltd., and the hs-TnT kit was provided by Shanghai Kalang Biotechnology Co. Ltd. All operations strictly followed the experimental standards.

### 2.5. Evaluation Indexes

The MMP-2 and hs-TnT levels in serum of the three groups, patients with different types of ACS, and patients with different numbers of diseased coronary vessels were compared and analyzed.

Adverse cardiovascular events included myocardial infarction, cardiac arrest, sudden cardiac death, and angina.

### 2.6. Statistical Methods

SPSS 21.0 statistical software was adopted to process the clinical data of the two groups, and the measurement data were expressed as ($\bar{x}\pm s$). The data between multiple groups were compared by one-way ANOVA and tested by *t*^2^. The enumeration data were expressed as [*n*(%)] and tested by *x*^2^, with statistically significant differences (*P* < 0.05).

## 3. Results

### 3.1. Comparison of Clinical Data of Patients in Each Group

The study results showed that the number of patients with smoking and drinking history in the acute group and the stable group was significantly higher than that in the control group (*P* < 0.05). The triglyceride levels in the acute group and the stable group were significantly higher than that in the control group (*P* < 0.05). The number of patients with hyperesteremia and hypertension in the acute group and the stable group was significantly higher than that in the control group (*P* < 0.05), as detailed in Table 1.

### 3.2. Comparison of hs-TnT and MMP-2 Levels of Three Groups of Experimental Subjects

The study results showed that the hs-TnT and MMP-2 levels in the acute group were significantly higher than those in the stable group and the control group and the hs-TnT and MMP-2 levels in the stable group were significantly higher than those in the control group, with statistically significant differences (*P* < 0.05), as detailed in Figures 1 and 2.

### 3.3. Comparison of the Incidence of Adverse Cardiovascular Events between the Two Groups after 30 Days

The study results showed that the incidence of cardiovascular events after 30 days in the acute group was significantly higher than that in the stable group, with statistically significant differences (*P* < 0.05), as detailed in Table 2.

### 3.4. Comparison of the hs-TnT and MMP-2 Levels in Patients with Different Types of ACS

The study results showed that the hs-TnT and MMP-2 levels in the AMI group were significantly higher than those in the UAP group, with statistically significant differences (*P* < 0.01), as detailed in Table 3.

### 3.5. Comparison of the hs-TnT and MMP-2 Levels in Patients with Different Numbers of Diseased Coronary Vessels

The study results showed that the hs-TnT and MMP-2 levels in the non-single-vessel group were significantly higher than those in the single-vessel group, with statistically significant differences (*P* < 0.05), as detailed in Table 4.

## 4. Discussion

ACS is mainly characterized by acute onset, severe illness, and high mortality. According to the survey results of the World Health Organization, about 15 million people worldwide die from cardiovascular and cerebrovascular diseases every year and more than half of them die from ACS [8]. With the change of daily lifestyle, the patients with ACS in China are on the rise year by year. It has become a consensus that early diagnosis and treatment can save more patients' lives. The cardiovascular biomarker is a kind of biochemical substance associated with the generation, development, diagnosis, clinical treatment, prognosis, and rehabilitation of patients' diseases, which is of great significance for disease treatment, diagnosis, and prevention. The sensitivity of hs-TnT is higher than that of cardiac troponin I (cTn I) and cardiac troponin T (cTn T) which are currently widely used as diagnostic biomarkers for myocardial injury caused by ischemic heart diseases in clinical and forensic medicine.

With the application of hs-TnT in the study, the increase of the hs-TnT level in patients with ACS can be measured at the time of onset and visit, which plays an important role in disease diagnosis. A large number of studies have shown that hs-TnT is a more common troponin [10], which only exists in human myocardium. When myocardial injury occurs in patients, the level of troponin concentration will show a rising trend, which is long lasting and the earliest increasing indicator in various physical indicators of patients. Therefore, this indicator can be used for the diagnosis and treatment of myocardial injury [11]. hs-TnT is also a sensitive inflammatory indicator which is synthesized by the liver and can effectively reflect the systemic inflammation of patients. Inflammation will occur in the rupture of plaque. The coagulation mechanism is affected by cytokines, which stimulates the human liver, promotes the production of a large amount of hs-TnT, and releases hs-TnT in the blood. MMP-2 can be formed in human fibroblasts, endothelial cells, macrophages, and other cells and have a joint effect with calcium and zinc ions, having a degradation effect on the human extracellular matrix. Relevant information showed that [12] the MMP-2 level in serum is an important cytokine for judging the prognosis of ACS and can be used as an important parameter for clinical risk prediction. Additionally, the MMP-2 level in serum plays an important role in the early diagnosis and treatment of acute high-risk coronary syndrome and in identifying potential risk factors.

The study results are consistent with the results of the “*Application Value of Serum Hypersensitivity Troponin T and Myoglobin Detection in Acute Myocardial Infarction*” by Yimei and Weipeng [9]. Compared with those in the stable group, hs-TnT and MMP-2 levels in the acute group remarkably increased, with statistically significant differences (*P* < 0.05). In [13] and others' studies, the dynamic follow-up survey of patients with ACS showed that the incidence of adverse cardiovascular events was 28%, the hs-TnT in serum was 2.08 ± 0.29 ng/ml, and the MMP-2 in serum was 0.52 ± 0.17 ng/ml. Relevant foreign data [14] showed that the hs-TnT high expression level is positively correlated with cardiovascular disease. It has been fully demonstrated that the hs-TnT and MMP-2 high expression levels in serums of the patients with ACS can effectively predict poor prognosis and increased incidence of cardiovascular events. In addition, attention should be paid to the prevention of cardiovascular events in such patients at a later stage [15].

However, there are some limitation here. It was conducted on a relatively small number of participants; a large number of population should be included in the following study. Furthermore, we should investigate if hs-TnT and MMP-2 levels in experimental models are of clinical interest also in terms of their use as potential biomarkers of disease progression and potential predictors of treatment efficacy.

In conclusion, hs-TnT combined with MMP-2 is of great significance for the diagnosis, prognosis, and treatment of ACS, which can effectively reflect the condition of patients with coronary artery disease and accurately evaluate the clinical risk factors, providing data support for disease treatment and rehabilitation.

## Figures and Tables

**Figure 1:** Comparison of hs-TnT levels of three groups of experimental subjects. The abscissa represents the acute group, the stable group, and the control group, while the ordinate represents the hs-TnT level. As shown in Figure 1, the hs-TnT level was the highest in the acute group and the lowest in the control group. hs-TnT: hypersensitive troponin T.

**Figure 2:** Comparison of MMP-2 levels of three groups of experimental subjects. The abscissa represents the acute group, the stable group, and the control group, while the ordinate represents the MMP-2 level. As shown in Figure 2, the MMP-2 level was the highest in the acute group and the lowest in the control group. MMP-2: matrix metalloproteinase 2.

**Table 1:** Comparison of clinical data of patients in each group (*n* = 40).

Factors	Acute group	Stable group	Control group	*t*_1_^2^(*x*^2^)/*p*_1_	*t*_2_^2^(*x*^2^)/*p*_2_	*t*_3_^2^(*x*^2^)/*p*_3_
Age (years old)	53.27 ± 1.45	53.04 ± 1.38	52.85 ± 1.46	0.73/0.47	1.29/0.20	0.58/0.56
Course of disease (year)	3.05 ± 0.56	3.21 ± 0.63	/	1.20/0.23	/	/
Male/female (case)	19/21	18/22	20/20	0.015/0.90	0.11/0.74	0.20/0.65
Drinking (%)	55% (22/40)	50% (20/40)	7.5% (3/40)	0.20/0.65	21.00/0	17.64/0
Smoking (%)	52.5% (21/40)	47.5% (19/40)	5% (2/40)	0.20/0.66	22.03/0	22.03/0
Triglyceride (mmol/l)	2.05 ± 0.43	1.86 ± 0.26	0.92 ± 0.19	2.39/0.02	15.20/0	18.46/0
Hyperlipidemia (case)	22	19	0	0.45/0.50	30.34/0	24.92/0
Hypertension (case)	24	173	3	2.45/0.12	24.65/0	13.07/0

*t*_1_^2^(*x*^2^)/*p*_1_ represents a comparison between the acute group and the stable group. *t*_2_^2^(*x*^2^)/*p*_2_ represents a comparison between the acute group and the control group. *t*_3_^2^(*x*^2^)/*p*_3_ represents a comparison between the stable group and the control group.

**Table 2:** Comparison of the incidence of adverse cardiovascular events between the two groups after 30 days.

Group	*n*	Myocardial infarction	Cardiac arrest	Sudden cardiac death	Angina pectoris	Incidence
Acute group	40	7.5% (3/40)	10% (4/40)	7.5% (3/40)	10% (4/40)	32.5%
Stable group	40	0	2.5%(1/40)	0	5% (2/40)	7.5%
*x* ^2^		3.1117	1.920	2.051	0.721	8.669
*p*		0.077	0.166	0.152	0.396	0.003

**Table 3:** Comparison of the hs-TnT and MMP-2 levels in patients with different types of ACS.

Group	N	Hs-TnT (ng/ml)	MMP-2 (ng/ml)
AMI group	51	1.79 ± 0.32	0.52 ± 0.17
UAP group	29	0.48 ± 0.11	0.37 ± 0.13
*t*		21.292	4.113
*p*		<0.01	<0.01

hs-TnT: hypersensitive troponin T; AMI: acute myocardial infarction.

**Table 4:** Comparison of hs-TnT and MMP-2 levels in patients with different numbers of diseased coronary vessels.

Group	*n*	hs-TnT (ng/ml)	MMP-2 (ng/ml)
Single-vessel group	41	0.67 ± 0.18	0.27 ± 0.14
Non-single-vessel group	39	1.91 ± 0.37	0.54 ± 0.22
*t*		19.207	6.582
*p*		<0.01	<0.01

MMP-2:matrix metalloproteinase 2; hs-TnT: hypersensitive troponin T; UAP: unstable angina pectoris.

## Data Availability

The data used during the present study are available from the corresponding author upon reasonable request.
